# Tumor-specific Th2 responses inhibit growth of CT26 colon-cancer cells in mice via converting intratumor regulatory T cells to Th9 cells

**DOI:** 10.1038/srep10665

**Published:** 2015-06-02

**Authors:** Jiang-Qi Liu, Xing-Yong Li, Hai-Qiong Yu, Gui Yang, Zhi-Qiang Liu, Xiao-Rui Geng, Shuai Wang, Li-Hua Mo, Lu Zeng, Miao Zhao, Yun-Ting Fu, Hong-Zhi Sun, Zhi-Gang Liu, Ping-Chang Yang

**Affiliations:** 1 ENT Institute of Shenzhen University School of Medicine and Shenzhen Key Laboratory of Allergy & Immunology, 518060, China; 2 Department of Surgery, the First Hospital, Liaoning Medical University, Jinzhou, 100044, China; 3 Longgang Central Hospital, Shenzhen, 518116, China; 4 Brain Body Institute, McMaster University, Hamilton, ON, Canada L8N 4A6

## Abstract

The abnormality of immune regulation plays a critical role in the pathogenesis of cancer; the underlying mechanism has not been fully understood yet. This study aims to investigate the role of cancer specific T helper (Th)2 response in the inhibition of colon cancer (Cca) cell growth. The results showed that with Cca cell (CT26 cell) extracts as an antigen, the Cca-extract specific Th2 response was induced in the Cca-bearing mice. The Cca mass size was significantly reduced, or radically disappeared (5 out of 10; or 50%); the survival rate was markedly improved in mice immunized with Cca-extract, but not in those immunized with another tumor cell (U87 cell) extracts or to bovine serum albumin. The immunization with Cca-extract also induced Cca cell apoptosis and converted the intra-Cca Tregs to T helper (Th) 9 cells. In conclusion, Cca-specific Th2 responses inhibit Cca growth in a mouse model via inducing Cca cell apoptosis and converting intra-Cca Tregs to Th9 cells.

Under physiological environment, the sporadic cancer cells in the body can be recognized and eliminated by the immune surveillance^1^. The cytotoxic CD8^+^ T cells are the major cell population to kill cancer cells^2^. Other immune cells, including natural killer cells^3^, CD4^+^ T cells^4^ and macrophages^5^ also inhibit cancer cells. However, in specific circumstances, the cancer killer cells may be dysfunctional; such as the intratumor infiltrating regulatory T cells (Treg) are capable of suppressing most effector T cell activities to impair the anti-tumor mechanism in the body. Tumor cells may thus escape from the immune surveillance. On the other hand, a number of publications have shown evidence to inhibit Tregs does suppress tumor growth^6^,^7^. However, it has not established such an anti-tumor remedy in tumor clinic.

Published data indicate that the proinflammatory CD4^+^ T cells can inhibit cancer cells via releasing anti-tumor cytokines^8^,^9^. The combination of proinflammatory CD4^+^ T cell therapy and chemotherapy may reciprocally reinforce the anti-tumor therapy, but has not been fully explored yet. The proinflammatory CD4^+^ T cells include T helper (Th)1 cells, Th2 cells and Th17 cells; and a fraction of Th9 cells was also characterized^10^,^11^. Among the Th cells, it is controversial about the role of Th17 cells in tumor growth^12^,^13^. The anti-tumor role of Th1, Th2 and Th9 cells has been well recognized^14^,^15^,^16^. Thus, to deliberately create polarization of Th1, Th2 or Th9 cells have the potential to bring about or facilitate anti-tumor activities^14^,^15^,^16^.

The animal models of antigen-specific Th2 polarization have been well established. In one of the models, animals were immunized with antigens mixing with adjuvant alum, which can induce similar pathological changes of allergic disorders such as intestinal allergy^17^. To investigate the anti-tumor role of antigen specific Th2 polarization, we created a cancer mouse model by inoculating a mouse Cca cell line, WT-CT-26 cells, to mice. The mice were immunized with Cca-extract (Cca-extract was used as a Cca antigen) to induce a Cca specific Th2 response in the Cca-bearing mice. The results showed the Cca mass was dramatically reduced or radically removed by the Cca-specific Th2 response. The Cca specific CD4^+^ T cells efficiently induced Cca cell apoptosis and suppressed the intra-Cca Tregs in the Cca-bearing mice via converting the Tregs to Th9 cells.

## Results

### Characterization of Cca specific Th2 response in Cca-bearing mice

Following published procedures, we developed a Cca BALB/c mouse model. The Cca-bearing mice were treated with the protein extracts of the Cca cells (Cca-extract) mixing with alum (using as an adjuvant) in the procedures established in our laboratory. After sacrifice, specimens of the blood and spleens were collected to be analyzed for the Cca specific Th2 response. We firstly assessed the Cca specific CD4^+^ T cells in the spleens by CFSE-dilution assay. The results showed that cells from naïve mice showed less than 5% cell proliferation (Fig. 1A,F); in the presence of the Cca-extract, 47.9% CD4^+^ T cell proliferation was detected in the Cca-bearing mice immunized with Cca-extract (Fig. 1B,F); cells from Cca-bearing mice immunized with U87-extract (Fig. 1C,F), or BSA (Fig. 1D,F), or treated with alum (Fig. 1E,F) alone showed 4.69%, 5.79% and 4.10%, respectively (p > 0.05 as compared with Fig. 1A). The levels of serum Cca-extract-specific IgE and Th2 cytokines were in parallel to the Teff cell proliferation (Fig. 1G–I). The results indicate that a Cca-extract-specific Th2 response is induced in the Cca-bearing mice.

### Records of colon cancer growth in the course of induction of Th2 response

Two weeks after inoculation, the Cca mass was about 2 cm to 2.5 cm in diameter in the mice. After treating with the immunization, the Cca mass was disappeared in 5/10 (50%) mice and reduced the mass size to 0.5 cm to 1.5 cm in the rest of 5 mice. In contrast, the Cca mass did not disappear in any of the Cca-bearing mice treated with U87-extract, or BSA, or saline; instead, the Cca mass grew to 850-1000 mm^3^ at the time point of death (Fig. 2A). In a 50-day observation period, no mice died in the Cca-extract group; instead, tumor-bearing mice in the rest three groups died between day 30 and day 36 after the tumor inoculation (Fig. 2B). The data suggest that the immunization to Cca-extract inhibits Cca growth and increases the tumor-bearing mouse survival in an cancer-allergen specific manner.

### Cca specific CD4^+^ T cells induce colon cancer cell apoptosis

We next took insight into the mechanism by which the Cca-specific Th2 response inhibits Cca growth. The Cca tissue was processed for TUNEL staining. The results showed that about 38.6% apoptotic Cca cells were observed in the group immunized with Cca-extract/alum (Fig. 3A,F), which were significantly less in the groups immunized with U87-extract (Fig. 3B,F), BSA (Fig. 3C,F) or alum (Fig. 3D,F). The results implicate that the Cca-specific Th2 response induces Cca cell apoptosis. To strengthen the data, we isolated CD4^+^ CD25^+^ CD127^+^ T cells (CD4^+^ T cells, in short) from the spleen of the Cca-bearing mice after immunization. The CD4^+^ T cells were cultured with Cca cells (Cca cell line, WT-CT-26) for 3 days in the presence of DC and then analyzed by flow cytometry (Fig. 3G). The results showed that 2.5% Cca cell was apoptotic after culture with CD4^+^ T cells from naïve mice (Fig. 3H,N). The frequency of apoptotic Cca cells was significantly increased (63.2%) after cultured with the CD4^+^ T cells isolated from the Cca-bearing mice immunized with Cca-extract (Fig. 3I,N). The results also showed that the culture with CD4^+^ T cells isolated from Cca-bearing mice immunized with U87 (Fig. 3J,N) or BSA (Fig. 3K,N) did not increase the frequency of apoptotic Cca cells. The results confirm that the Cca-specific Th2 response can induce Cca cell apoptosis. To elucidate if the cell-cell contact is required in the induction of apoptosis, in separate experiments, Cca cells and the CD4^+^ T cells were cultured in separate chambers of Transwell system for 3 days. The results showed that the apoptosis was still induced in Cca cells (Fig. 3L,N), which indicates that the cell-cell contact is unnecessary in the induction of Cca cell apoptosis by the present experimental setting. To test if T cell-derived IL-9 played a role in the induction of apoptosis of Cca cells, we created Cca model in the IL-9-deficient mice, from which the CD4^+^ T cells were isolated and cultured with Cca cells and DCs as described above. The apoptosis of Cca cells was abolished (Fig. 3M,3N). The results implicate that the immunization with Cca extracts induces Cca-specific IL-9-producing T cells, which induce Cca cell apoptosis.

### Intra-Cca Tregs are inhibited by the colon cancer specific CD4^+^ T cells

Next we assessed the frequency of Tregs in Cca tissue of Cca-bearing mice. As shown by flow cytometry, Tregs were detected in the single cells of Cca tissue of mice (Fig. 4A,F) that were significantly less in the mice immunized with Cca-extract (Fig. 4B,F). The frequency of Tregs in Cca tissue of mice immunized with either U87-extract (Fig. 4C,F) or BSA (Fig. D, 4F) was similar to those Cca-bearing mice treated with alum. The results suggest that immunization with Cca-extract inhibits the intra-Cca Tregs, which does not occur when the Cca-bearing mice are immunized with other antigens.

In the flow cytometry data of Fig. 4A–D, we observed a fraction of CD4^+^ Foxp3^-^ cells with dramatic differences between groups. It was 8.4% in the Cca-extract-immunized Cca-bearing mice, 1.5%, 1.4% and 1.6% in the Cca-bearing mice immunized with U87-extract, BSA and alum respectively (Fig. 4A–E,G). Further analysis showed that the IL-9^+^ cells were detected in this fraction of CD4^+^ Foxp3^-^ T cells, which was significantly more in the Cca-bearing mice immunized with Cca-extracts as compared with the rest groups (Fig. 4H). The results indicate that Th9 cells (16) are generated in the Cca-bearing mice after immunization with Cca-extracts. To strengthen the data, a group of mice was received a neutralizing anti-IL-4 antibody, which blocked the immunization-reduced Foxp3^+^ Tregs and -generated Th9 cells in Cca-bearing mice (Fig. 4).

### Specific Th2 response converts intra-Cca Tregs to Th9 cells

Based on published data that Tregs may be converted into Th9 cells under given circumstances (16) and the data of Fig. 1, 2, 3, 4, we postulated that the Cca-specific Th2 response might convert Tregs to Th9 cells. To test the hypothesis, we isolated CD4^+^ CD25^+^ CD127^−^ Tregs from Cca tissue or naïve mouse spleen, labeled with CFSE and cultured with CD4^+^ CD25^+^ CD127^+^ T cells (isolated from the spleens of Cca-bearing mice, or from naïve mice) for 6 days in the presence of Cca-extract and DC. The cells were analyzed by flow cytometry. The results showed that the CFSE was still detectable in the Tregs at the end of culture (Fig. 5A). The gated CFSE^+^ cells in Fig. 5A were further analyzed. About 83% Tregs from Cca tissue were converted to IL-9^+^ cells (Fig. 5B); only 1.5% naïve Tregs were converted to IL-9^+^ cells (Fig. 5C); the conversion was abolished by the presence of a neutralizing anti-IL-4 (Fig. 5D) or anti-TGF-β (Fig. 5E) antibody. The results implicate that the CD4^+^ T cell-derived IL-4 collaborates with TGF-β in Tregs to convert Tregs to Th9 cells in a Cca-extract-dependent manner. To strengthen the data, in separate experiments, U87-extract (Fig. 5F) or BSA (Fig. 5G) was added to the culture instead of Cca-extract. The results showed none of the Tregs was converted to Th9 cells. On the other hand, the presence of rIL-4 converted Cca-derived Tregs and naïve Tregs to Th9 cells (Fig. 5H).

To strengthen the data of Fig. 5, we created a Cca model with Ly5.1 and Ly5.2 mice. Tregs were isolated from the Cca tissue of Ly5.2 mice. On day 1 of immunization, the Ly5.2 Tregs were adoptively transferred to Ly5.1 Cca-bearing mice. The mice were sacrificed on day 14; the Cca tissue was excised; single cells were prepared and analyzed by flow cytometry. The results showed that about 2-3% Ly5.2 cells were detected in the single cells of Cca tissue (Fig. 6A–E); more than 90% of Ly5.2 cells were still Foxp3^+^ in the Cca-bearing mice treated with saline (Fig. 6F,J). The Ly5.2 Tregs were converted to IL-9^+^ Foxp3^−^ Th9 cells in the mice immunized with Cca extracts (Fig. 6G,J). To elucidate if the conversion was Cca antigen specific, with the same procedures above, we replaced the Cca extracts with BSA. The results showed that the conversion of Ly5.2 Tregs to Ly5.2 Th9 cells was abolished (Fig. 6H,J). In addition, treatment with a neutralizing anti-IL-4 antibody also inhibited the conversion of Tregs to Th9 cells (Fig. 6I,J).

## Discussion

Although the tumor research advanced rapidly in the last several decades, the tumor-induced death is still the largest threatening factor in human life. The therapeutic effect of tumor is to be further improved. The present study has revealed that the induction of a cancer specific immune response can suppress Cca cell growth, which may have the therapeutic potential in the treatment of Cca.

The induction of antigen specific immune response in animal models has been employed in the research of a number of diseases, such as asthma, allergic rhinitis and dermatitis. The key parameters of antigen specific Th2 response include higher levels of serum antigen specific IgE, IL-4, IL-5 and IL-13, and antigen-specific T cell proliferation. The present data show that after immunization with Cca extracts, high levels of Th2 cytokines and Cca-specific IgE were detected in the serum; the Cca-extract-specific CD4^+^ T cell proliferation was also detected. Thus, the antigen specific Th2 response is not only induced in naïve animals, but also can be induced in tumor-bearing mice using cancer extracted proteins as a specific antigen.

The Cca-extract using in the present study is a mixture of proteins extracted from Cca cells. Similar strategies are also employed in some other animal models of Th2 polarization; such as using peanut extracts to create food allergy animal models^18^ and using mite extracts to create asthma animal models^19^; these antigens are also a mixture of peanut extracts or a mixture of mite extracts. Antigen-specific Th2 polarization can be induced using these mixtures of antigens.

Our results show that after immunization, the Cca mass size was markedly reduced, indicating that the immunization inhibits Cca cell growth in the mice. The reduction of Cca mass implicates the number of Cca cell is reduced in the immunized mice. The inference is supported by further experimental results. We observed the Cca cell apoptosis in the mice immunized with Cca-extracts. To induce cancer cell apoptosis is the principal mechanism in a number of anti-cancer therapeutics; such as radiotherapy^20^ and some anti-cancer drugs^21^. Our study provides a novel remedy for the anti-cancer therapeutics by showing that the induction of a cancer-specific Th2 response also induces cancer cell apoptosis. It is noteworthy to elucidate that the inhibitory effect on cancer cell growth in the present study is cancer-specific as we only observed the inhibitory effect in Cca-bearing mice immunized with Cca-extract, but not in those mice immunized with U87-extract or BSA.

It is proposed that the intratumor Tregs play a critical role in compromising the anti-tumor mechanism in the body. Such as Wang *et al.* indicate that the tumor specific Tregs suppress tumor specific CD8^+^ T cells^22^. Our data also show a large number of Tregs in the Cca tissue. This is in line with the reports of other investigators; such as Wu *et al.* suggest that the intra-gastric cancer Tregs have multiple suppressive effect on other immune cells^23^. Our data also show that after immunization with Cca-extracts, the frequency of intra-Cca Tregs reduced markedly. Our previous studies also show that the frequency of Tregs is significantly reduced after immunization in food allergy mouse models^24^. Since intra-tumor Tregs play a critical role in compromising the anti-tumor immunity, to inhibit Treg function or reduce Treg number can inhibit tumor growth^6^,^7^, the present data suggest that to induce Cca-specific Th2 polarization may be operative to inhibit the intra-Cca Tregs. The inference is supported by the present data that, after immunization with Cca-extract, the Cca mass size is markedly reduced.

The results also show that the Th2 polarization converts intra-Cca Tregs to Th9 cells, in which IL-4 plays a critical role. The results are in line with published data, Cardalhon *et al.* indicate that IL-4 converts Tregs to IL-9 and IL-10 production cells^25^; Th9 cells are a fraction of anti-tumor cells^16^. Taken together, the present data indicate that the Cca-specific Th2 response can be induced in Cca-bearing mice. The Cca-specific Th2 response can induce Cca cell apoptosis and convert intra-Cca Tregs to Th9 cells, and thus, suppress Cca growth.

## Materials and methods

### Reagents

The fluorochrome-labeled antibodies of CD4, Foxp3 and IL-9 were purchased from BD Biosciences (Shanghai, China). The ELISA kits of IL-4, IL-5, IL-13, IFN-γ, IgE, terminal deoxynucleotidyltransferased dUTP nick end labeling (TUNEL) kit, neutralizing anti-IL-4 and anti-TGF-β were purchased from R&D Systems (Shanghai, China). The Annexin V kit was purchased from Sigma Aldrich (Shanghai, China). The immune cell isolation kits were purchased from Myltenyi Biotech (Guangzhou, China). The anti-Ly5.2 antibody was purchased from Santa Cruz Biotech (Santa Cruz, CA).

### Mice

The animal study procedures were approved by the Animal Ethic Committee at Shenzhen University. The experiments were done in accordance to the guidelines. Male BALB/c mice (8-10 week old) were purchased from Guangdong Experimental Animal Center. The IL-9-deficient mice, Ly5.1 and Ly5.2 mice were purchased from Jackson Laboratory (Harbor, Maine). The mice were maintained in a pathogen free environment with access to food and water freely.

### Cca cell culture

A mouse Cca cell line (WT-CT-26 cells) was purchased from ATCC (Manassas, VA) and cultured in RPMI1640 medium supplemented with 10% fetal bovine serum, 100 U/ml penicillin, 0.1 mg/ml streptomycin and 2 mM L-glutamine. The medium was changed in 1-2 days. The cell viability was 98.5% as assessed by the Trypan exclusion assay.

### Cca cell inoculation

Cca cells were cultured to confluence and suspended in PBS, and were injected into the subcutaneous space of the groin at 10^6^ cells/mouse.

### Preparation of cancer cell extracts (Cca-extract and U87-extract)

WT-CT-26 cells or U87 cells (a glioma cell line using as a control cancer cell line) were lysed by a lysis buffer. The protein levels of the extracts were determined by the Bio-Rad protein assay.

### Immunization of Cca-bearing mice

After the Cca mass grew to 2 cm in diameter (measured with a vernier caliper), each mouse was injected subcutaneously at back skin with 0.5 mg Cca-extract mixing in 0.3 ml alum on day 0 and day 3. The mice were challenged with 0.5 mg Cca-extract by intraperitoneal injection on day 5, 7, 9, 11 and 13 respectively. A portion of the mice was sacrificed on day 14 to determine the Th2 response. The blood and Cca mass were collected for further experiments. Control Cca-bearing mice were treated with U87-extract/alum, or BSA/alum, or alum alone. To block the role of IL-4, recipient mice were received a neutralizing anti-IL-4 antibody (i.p.) at 0.25 mg/mouse on day 7 and day 10 respectively.

### Immune cell isolation

The spleens and Cca tissue were collected from mice upon sacrifice. Single cells were made from the spleens and Cca tissue with the established procedures of our laboratory^22^,^26^. Immune cells were isolated from the single cells by magnetic cell sorting with commercial reagent kits. The purity of each cell type was greater than 98% as assessed by flow cytometry following our established procedures^27^.

### Assessment of Cca-specific CD4^+^ T cell response

The Cca-specific T cell response was assessed by carboxyfluorescein succinimidyl ester (CFSE)-dilution assay. CD4^+^ CD25^−^ T cells (labeled with CFSE) and dendritic cells (DC) were cultured at a ratio of 5:1 in the presence of Cca-extract, or U87-extract, or BSA, at a concentration of 10 μg/ml. The cells were collected after 3 days and analyzed by flow cytometry. The culture supernatant was collected and analyzed by ELISA. The proliferation of T cells and the levels of IL-4 were recorded and regarded as the indicators of the Cca-specific Th2 response.

### Enzyme-linked immunosorbent assay (ELISA)

The levels of cytokines of IL-4, IL-5, IL-13 and IFN-γ were determined by ELISA with commercial reagent kits following the manufacturer’s instructions. The serum levels of Cca-specific IgE were determined by an in-house ELISA. Briefly, the serum was diluted 10 folds; the microplate wells were coated with the diluted serum (or BSA using as a control) at 20 μg protein/ml; the plates were placed at 4 °C overnight. The wells were blocked by 1% BSA for 30 min at room temperature. A primary anti-IgE monoclonal antibody (1:2000) was added to each well; the plates were incubated at room temperature for 1 h; after washing with PBST for 3 times, a secondary antibody (conjugated with horseradish peroxidase) was added to each well, and incubated for 1 h at room temperature. After washing with PBST, 0.1 ml 3,3’,5,5’-Tetramethylbenzidine substrate was added to each well; the reaction was stopped by adding 50 μl 2N H_2_SO_4_. The plates were read with a microplate Reader (HTS Multi-Mode, BioTek, Guangzhou, China) at 450 nm. The data of sample wells were normalized by subtracting the readout of the BSA wells (negative control). All samples were tested in triplicate; an average of data from three wells was used as one datum.

### *In situ* apoptosis assessment

The apoptotic cells in the Cca tissue sections were stained with a TUNEL reagent kit following the manufacturer’s instructions. The positively stained cells were counted in 30 randomly selected fields under a light microscope. The slides were coded; the observers were not aware of the codes to void the observer bias.

### Induction of Cca cell apoptosis by culturing with Cca-specific CD4^+^ CD25^+^ CD127^+^ T cells

CD4^+^ CD25^+^ CD127^+^ T cells were isolated from the spleens of mice with or without Cca. The CD4^+^ CD25^+^ CD127^+^ T cells were cultured with Cca cells (WT-CT-26 cells) at a ratio of 1:2 (T cell:Cca cell) for 3 days in the presence of dendritic cells (CD11c^+^ DC) (DC:T cell = 1:10). Cca-extract, or U87-extract, or BSA was added to the culture at a dose of 10 μg/ml. The cells were collected at the end of culture, and stained with antibodies of CD4, CD11c, propidium iodide and Annexin V reagent following the manufacturer’s instructions, and analyzed by flow cytometry. The CD4^+^ T cells and CD11c^+^ DCs were gated out first; the remaining Cca cells were further analyzed for the frequency of apoptotic cells.

### Flow cytometry

Cells were fixed with 2% paraformaldehyde containing 0.1% Triton X-100 for 2 h. After washing with PBS, the cells were blocked with 1% BSA for 30 min and followed by incubating with fluorochrome-labeled antibodies at concentrations of 100 ng-500 ng/ml for 1 h at room temperature. After washing, the cells were analyzed with a flow cytometer (FACSCanto II, BD Biosciences, Shanghai, China).

### Statistics

The data were presented as mean ± SD. Differences between groups were determined by ANOVA. A p < 0.05 was set as a significant criterion.

## Additional Information

**How to cite this article**: Liu, J.-Q. *et al.* Tumor-specific Th2 responses inhibit growth of CT26 colon-cancer cells in mice via converting intratumor regulatory T cells to Th9 cells. *Sci. Rep.* **5**, 10665; doi: 10.1038/srep10665 (2015).

## Figures and Tables

**Figure 1:** Cca-specific Th2 response in mice. The treatment of Cca-bearing BALB/c mice was denoted above the flow cytometry histograms. Teff cells (labeled with CFSE) and DCs (T cell:DC = 5:1) were isolated from the spleens and cultured in the presence of Cca-e (10 μg/ml) for 3 days. **A**–**E**, the histograms indicate the proliferation of the Teff cells. **F**, the bars indicate the summarized data of **A**–**E**. **G**–**I**, assessed by ELISA, the bars indicate the levels of cytokines in the culture supernatant of **A**–**E** (**G**), the serum specific IgE and IgG of the mouse groups **A**–**E** (**H**), and the serum Th2 cytokine levels of the mouse groups **A**–**E** (**I**). The data of **F**–**I** are presented as mean ± SD. *, p < 0.01, compared with group **A**. Each group consisted of 10 mice. The data are representatives of 10 independent experiments.

**Figure 2:** Effect of specific treatment on Cca mass size and weight. A–D, Cca**-**bearing mice were treated with Cca-e (extract)/alum, or U87-e/alum, or BSA/alum, or saline/alum. Cca mass was measured from day 3 to day 27. **A**, the curves indicate the tumor size on day 27. **B**, the curves indicate the survival rate of the tumor bearing mice. Each group consists of 10 mice. *, p < 0.01, compared with the saline group.

**Figure 3:** Assessment of Cca cell apoptosis. **A**–**E**, Cca tissue was excised from the Cca-bearing mice after treatment (as denoted above each image) and processed the cryosections for TUNEL staining. The images show the apoptotic cells (stained in brown). **F**, the bars indicate the frequency of apoptotic cells averaged from 30 fields/sample. **G**, CD4^+^ CD25^+^ CD127^+^ T cells (in short, CD4^+^ T cells) were isolated from the excised Cca tissue and cultured with Cca cells (at a ratio of 1:1) for 3 days in the presence of CD11c^+^ DC. The gated cells are Cca cells (WT-CT-210 cells) and were further analyzed by flow cytometry. **H**–**L**, the gated cells indicate Annexin V^+^ and propidium iodide (PI)^+^ apoptotic cells. The sources of samples are denoted above each subpanel. Cca-e/Alum-a: The experiments were done in Transwell system. Cca-e/Alum/b: CD4^+^ T cells were isolated from Cca-bearing IL-9-deficient mice. **N**, the bars indicate the summarized data of apoptotic cells of panels **H**–**L**. The data of bars in F and M are presented as mean ± SD. *, p < 0.01, compared with **A** (**F**), or **H** (**M**). The data are representatives of 3 independent experiments.

**Figure 4:** Cca-specific Th2 response inhibits Tregs in Cca tissue. Cca-bearing mice were treated as denoted above each dot plot panel of **A**–**E**. Cca tissue was excised from the mice and processed for single cells and analyzed by flow cytometry. **A**–**E**, the dot plots indicate the frequency of CD4^+^ or/and Foxp3^+^ cells. **F**, the bars indicate the summarized frequency of Tregs in gate 1 (G1) of A–E. G–H, the bars indicate the summarized CD4^+^ Foxp3^-^ cell frequency (**G**) and IL^-^9^+^ cell frequency (**H**) in gate 2 (G2) of **A**–**E**. Ab: Mice were received a neutralizing anti-IL-4 antibody. The data of bars are presented as mean ± SD. *, p < 0.01, compared with group **A**. Each group consisted of 10 mice. The data are representatives of 10 independent experiments.

**Figure 5:** Cca-specific Th2 response converts intra-Cca Tregs to Th9 cells. CD4^+^ CD25^+^ CD127^+^ T cells and DCs were isolated from mice sensitized to Cca-e or U87-e. Intra-Cca Tregs were isolated from Cca-tissue and labeled with CFSE. CD4^+^ T cells and Tregs were cultured at a ratio of 1:1 in the presence of DCs, Cca-e (or U87-e, or BSA) (10 μg/ml) and IL-2 (10 ng/ml) for 10 days. The additional treatment is denoted above each subpanel. The cells were collected and stained with an anti-IL-9 antibody, and analyzed by flow cytometry. **A**, the gated dot plots indicate CFSE^+^ cells. **B**–**H**, the histograms indicate the frequency of IL-9^+^ cells in the gated cells of **A**. **I**, the bars indicate the summarized data of **B**–**H**. The data of bars are presented as mean ± SD. *, p < 0.01, compared with group **B**. Each group consists of 10 mice. The data are representatives of 10 independent experiments.

**Figure 6:** Cca-specific immune response converts Tregs to Th9 cells in Cca-bearing mice. A Cca model was created with Ly5.1 and Ly5.2 mice. The Cca-bearing mice were immunized with Cca extracts. CD4^+^ CD25^+^ CD127^−^ Tregs were isolated from Ly5.2 mice by MACS (purity >98%) and transferred to Cca-bearing Ly5.1 mice on the day of immunization at 10^6^ cells/mouse via tail vein injection. The mice were sacrificed on day 14. Single cells were prepared from the excised Cca tissue and analyzed by flow cytometry. **A**–**D**, the gated dot plots indicate the frequency of Ly5.2 cells. **E**, the bars indicate the summarized data of **A**–**D**. **F**–**I**, the dot plots indicate the frequency of Foxp3^+^ Tregs and IL-9^+^ cells. **J**, the bars indicate the summarized data of **F**–**I**. The data of bars are presented as mean ± SD. *, p < 0.01, compared with group **A**. Each group consisted of 6 mice. Samples from individual mice were processed separately. The data are representatives of 6 independent experiments.
